# Efficacy and Clinical Value of Negative-Pressure Wound Therapy with Instillation (NPWTi) of Compound Phellodendron Liquid in the Treatment of Diabetic Foot Ulcer: A Prospective Cohort Study

**DOI:** 10.1155/2022/7540020

**Published:** 2022-08-09

**Authors:** Yang Zhao, Xiaohong Dai, Yan Sun, Weixiang Liao, Yan Peng, Jiuyi Yang

**Affiliations:** ^1^Department of Peripheral Vascular (Wound Repair), Chongqing Traditional Chinese Medicine Hospital, Chongqing 400021, China; ^2^Department of Urology, Chongqing Traditional Chinese Medicine Hospital, Chongqing 400021, China

## Abstract

**Objective:**

To evaluate the efficacy and application value of compound Phellodendron liquid (CPL) for negative-pressure wound therapy with instillation (NPWTi) in the treatment of diabetic foot ulcers by observing the improvement of diabetic foot ulcers.

**Methods:**

Sixty patients with diabetic foot ulcers who met the inclusion criteria were admitted to the Department of Peripheral Blood Vessels (Wound Repair) of Chongqing Hospital of Traditional Chinese Medicine from August 2020 to August 2021. The random number table method divided it into the CPL NPWTi group and normal saline NPWTi group, with 30 cases in each group. The experimental group adopted FufangHuangbaiye for NPWTi, and the control group used normal saline for NPWTi. The treatment effect was evaluated by baseline index, wound healing observation index, inflammatory factor index, pain scores during dressing change, and the number of days in hospital.

**Results:**

After 10 days of treatment, the symptom integration, procalcitonin (PCT), and C reactive protein (CRP) of the CPL NPWTi group were significantly reduced compared with the normal saline NPWTi group, while there was no obvious difference between wound area and erythrocyte sedimentation rate (ESR). The wound area, symptom integral, PCT, ESR, and CRP of the CPL NPWTi group were significantly reduced compared with the normal saline NPWTi group after treatment for 20 days and 30 days. The positive proportion of bacterial culture in the CPL NPWTi group was significantly reduced compared with the normal saline NPWTi group after treatment for 10 days, 20 days, and 30 days. After treatment, the pain scores during dressing change and the number of days in hospital in normal saline NPWTi group were significantly lower than those in the CPL NPWTi group.

**Conclusion:**

Compound Phellodendron liquid NPWTi therapy can improve diabetic foot ulcers, providing a safe and effective method for treating diabetic foot ulcers.

## 1. Introduction

A diabetic foot is a lesion of foot ulcers or deep tissue destruction caused by factors such as peripheral neuropathy, peripheral vascular disease, and infection, which can easily lead to severe complications such as disability and even death [1]. Among them, diabetic foot infection (DFI) accounts for 40% to 80% of diabetic foot patients, and the degree of infection affects the prognosis of patients, which is one of the main causes of amputation and death in diabetic patients [2]. Studies have reported that 5% to 10% of patients with diabetes mellitus have some degree of diabetic foot ulcers, and 1% of those need amputation [3]. Approximately 85% of nontraumatic lower-limb amputations are caused by diabetic foot; the rate of reamputation in the 5 years after amputation is as high as 50%, and the mortality rate is as high as 70% [4–6]. Infection is one of the essential factors in the nonhealing of diabetic foot wounds. Bacteria can cause an inflammatory response that prompts the body to secrete harmful cytokines, causing blood vessels to contract and inhibiting tissue cell growth. Bacteria and other microbes also hinder wound healing by increasing metabolism to ingest nutrients and oxygen needed for tissue repair and growth [6]. Negative pressure wound aspiration therapy provides a moist healing environment for wounds, promotes rapid epithelialization of wounds, stimulates angiogenesis, increases blood transport to wounds, aspirates exudates, reduces edema, and promotes granulation tissue growth [7], thereby promoting healing of diabetic foot wounds. However, infection is one of the contraindications to suction therapy for negative pressure wounds [8]. Negative pressure wound therapy with instillation (NPWTi) is a new type of wound treatment method, alternately combining negative pressure wound suction treatment with liquid perfusion for treatment. The secretions and necrotic tissue of the wound tissue are better drained, and the local bacterial load is reduced by intermittently cleaning the wound surface with fluid. Wound aspiration therapy with less negative pressure can significantly reduce the bacterial load on diabetic foot wounds [9]. Clinical trials have demonstrated that NPWTi effectively promotes DFI wound healing [10]. At present, common drip irrigation solutions mainly include normal saline, biguanide fungicides, silver nitrate, 1% povidone-iodine, antibiotics, and insulin [11]. Still, there is no report on the choice of the best drip irrigation solution and Chinese medicine drip irrigation solution. FufangHuangbaiye is a compound water-like topical preparation formed by forsythia, golden cypress, dandelion, honeysuckle, centipede, and other traditional Chinese medicine ratios. Forsythia can disperse pus and detoxify heat; detoxification and golden cypress can detoxify and heal sores, clear heat, dry, and wet. They are a principal drug. Dandelion and honeysuckle are used as adjuvant drugs, which can enhance the effect of forsythia and golden cypress in draining pus and detoxification. Centipedes can reduce inflammation and cure sores, attack poison, and scatter knots. The combination of various drugs can synergistically reduce swelling and pain, remove saprophytic muscles, and clear heat and detoxify. Modern pharmacological studies have shown that FufangHuangbaiye has anti-infection and anti-inflammatory effects, which promote angiogenesis, alleviate inflammatory symptoms, eliminate incisional redness and swelling, and accelerate wound healing. The drug can be directly entered into the deep tendon space and pus cavity through topical treatment, which is conducive to removing wound pathogens, controlling and preventing infection, and promoting autolysis of necrotic tissue [12]. Traditional Chinese medicine preparation compound Phellodendron liquid (CPL) is an effective treatment method for DFI. In order to improve the drainage effect, reduce the infection rate of the wound, and shorten the wound healing time, this study used the closed negative pressure suction technique combined with the compound cork liquid coating intermittent irrigation to treat the diabetic foot ulcer Wagner grade 2-3 and observed its clinical treatment effect, thus providing a reference for clinical treatment.

## 2. Information and Methods

### 2.1. General Information

From August 2020 to August 2021, 60 patients with diabetic foot ulcers who met the inclusion criteria were admitted to the Department of Peripheral Vascular (Wound Repair) of Chongqing Hospital of Traditional Chinese Medicine. The random number table method divided it into the CPL NPWTi group and normal saline NPWTi group, with 30 cases in each group. There was no statistically significant difference in the comparison of basic data such as age and sex between the two groups (*P* > 0.05), which was comparable (Table 1). This trial is conducted by the Helsinki Declaration (2000 Edition) and China's relevant norms and regulations for clinical trial research. No patients dropped out of treatment.

### 2.2. Inclusion Criteria

1. *Diabetic Foot Ulcer (DFU)*. Those who meet the Western medical diagnostic criteria of DFU in the minutes of the 2013 China Forum on Diabetic Foot and Related Diseases [13], it meets the TCM diagnostic criteria of DFU in the Guidelines for Clinical Research of New Drugs in Chinese Medicines [14]; it is diagnosed as damp heat toxicity; the main symptom is ulcer; the secondary symptom is yellow urine, dry stool, thirst, pain, and burning around the sores. The tongue veins are lichen yellow, tongue redness, and pulse number, of which the secondary symptoms meet at least 2 items, the main symptoms are necessary, and the reference to the tongue pulse can be diagnosed
2. Age 50 to 85 years old
3. Ankle-brachial index 0.7 ~ 1.2
4. DFU Wagner clinical grades 2 to 3
5. Wound nonhealing ≥2 weeks and meets the diagnostic criteria for chronic wounds
6. Positive bacterial culture results
7. Hemoglobin > 100 g/L
8. Communicate with patients and their families to obtain cooperation and sign informed consent forms

### 2.3. Exclusion Criteria

1. After debridement, the tissue is brittle, easy to bleed to the touch, the bleeding is difficult to stop or the coagulation function is impaired, and NPWTi treatment cannot be carried out immediately
2. The wound is painful and cannot tolerate NPWTi treatment
3. Simultaneous concomitant infection of other important organs, such as respiratory tract and urinary tract infections
4. With severe liver and kidney disease, cardiovascular disease, blood disease, or malignancy. Patients with severe impairment of liver and kidney function
5. Local necrosis is severe and requires amputation surgery
6. Patients with incomplete clinical data

### 2.4. Termination or Shedding Criteria

1. Patients who die during the experiment or whose family members voluntarily give up and sign for discharge
2. Study of patients who were transferred to other departments for less than 7 days
3. Other adjuvant therapies that significantly impacted trial results were received during the study

### 2.5. Treatment

1. *Basal Treatment*. Systematic basic medical treatment is provided to all patients, including smoking cessation and alcohol restriction, diabetic diet, and control of blood pressure, blood glucose, and lipid levels. While awaiting the results of bacterial culture, antibiotic regimens are empirically selected based on the severity of the patient's foot infection and possible pathogens, and a final anti-infection regimen is developed based on the results of bacterial cultures and drug susceptibility tests. Patients are debridement before treatment, removing heavily infected, inactivated tissue, expanding deep pus and sinus tracts, and maximizing the preservation of incompletely inactivated tissue from the wound. The wound is carefully evaluated each time the dressing is changed, and if the wound is infected or necrotic, debridement should be carried out promptly
2. *Group Therapy*. The random number table method was used to randomly divide 60 patients into 2 groups, each group of 30 cases, the experimental group adopted FufangHuangbaiye (Shandong Hanfang Pharmaceutical Company) for NPWTi, and the control group used normal saline NPWTi. The negative pressure device adopts a central negative pressure. The course of treatment was the same in both groups. After debridement, trim the appropriate foam dressing according to the size of the wound (Shandong Weigao Xinsheng Medical Equipment Co., Ltd.) and place it on the wound bed. After 5% of the iodine is disinfected to the normal skin around the ulcer surface, it is sealed with a semipermeable film. The negative pressure suction tube and the liquid delivery tube are connected to the negative pressure equipment. The CPL or normal saline is connected to the solution delivery pipe as the drip irrigation solution. The amount of liquid depends on the size of the wound surface, which can be fully impregnated with the wound surface and does not cause the negative pressure sealing film to soak in moisture leakage due to excessive liquid amount, and about 1 ml of drip irrigation solution is required per square centimeter wound surface. The negative pressure selects the continuous mode. The pressure is set to 100-400 mmhg according to the wound situation. The drip irrigation solution is adjusted to 15 drops per minute, and the negative pressure rapid drip irrigation is suspended every 8 hours for the negative pressure 15-20 ml, every 7 days for a treatment cycle

### 2.6. Indicator

1. Baseline data

The sex, age, height, weight, blood glucose level, and comorbid diseases of the two groups of patients were collected.

(2) Observational indicators of wound healing

We conducted a 30-day follow-up study of the patients and looked at the specifics of the patients. The area of diabetic foot wounds in the two groups before treatment and after treatment 10 d/20 d/30 d, as well as the observation of the change of diabetic foot wound symptom scores, is recorded, and the quantitative table of diabetic foot symptoms is shown in Table 2.

(3) Indicators of inflammatory factors before and after treatment

Procalcitonin (PCT), erythrocyte sedimentation rate (ESR), and C-reactive protein (CRP) are detected. The wound is cultured with secretion bacteria.

(4) Patient condition evaluation

Pain scores during dressing change and the number of days in hospital.

### 2.7. Statistical Analysis

The experimental data analysis was based on SPSS20.0 statistical software. The measurement data were expressed as mean ± standard deviation (^−^*x* ± *s*). The two sets of metrological data were compared with the *t*-test, and the counting data were represented by [*n*(%)], *X*^2^ test was performed, and *P* < 0.05 was statistically significant for the difference.

## 3. Results

### 3.1. Wound Area and Symptom Integral

Before the treatment, there was no significant difference in the wound area and symptom integral between the CPL NPWTi group and the normal saline NPWTi group. After 10 days of treatment, the symptom scores of the CPL NPWTi group were significantly reduced compared with the normal saline NPWTi group, while the wound area was not significantly different. The wound area and symptom scores of the CPL NPWTi group were significantly reduced compared with normal saline NPWTi group after 20 days and 30 days of treatment (Table 3, Figure 1).

### 3.2. Indicators of Inflammatory Factors before and after Treatment

After 10 days of treatment, the PCT and CRP of the CPL NPWTi group were significantly reduced compared with the normal saline NPWTi group, while the ESR did not change significantly. After treatment for 20 and 30 days, the differences in PCT, ESR, and CRP in the CPL NPWTi group were statistically significant compared with the normal saline NPWTi group (Table 4 and Figure 2).

### 3.3. Wound Secretion Bacterial Culture Results

After treatment, the positive proportion of bacterial cultures in both groups decreased, and after 10, 20, and 30 days of treatment, the positive proportion of bacterial cultures in the FufangHuangbaiye NPWTi group was significantly reduced compared with the normal saline NPWTi group (Table 5).

### 3.4. The Number of Days in Hospital and Pain Scores during Dressing Change Results

After treatment, the pain scores during dressing change and the number of days in hospital in normal saline NPWTi group were significantly lower than those in the CPL NPWTi group, and the difference was statistically significant, see Table 6.

## 4. Discussion

Chinese medicine believes diabetic foot ulcers belong to the category of “gangrene,” mostly based on blood stasis block, choroidal obstruction due to wet injection or hot poison knots, and disease. The wound is often red and swollen and is often accompanied by fever, severe pain, odor, increased pus, and secretions. To reduce swelling and dispel decay, detoxification, loose knots, and communication as the treatment rules, the treatment is divided into internal treatment and external treatment, and external treatment is the emphasis of surgery. CPL is composed of golden cypress, forsythia, honeysuckle, dandelion, centipede, etc., which has the function of clearing heat, detoxification, swelling, and decay. It is used to treat osteomyelitis, ulcer ulceration, trauma infection, and so on. CPL can significantly promote the healing of skin wounds and has obvious inhibitory effects on Staphylococcus aureus, Streptococcus beta, and Pseudomonas aeruginosa [15]. Modern pharmacological studies have shown that CPL can reduce the expression of IL-1*β* and increase the expression of the growth factor transforming growth factor-*β* (TGF-*β*). Its activation of nuclear factor erythroid 2-related factor 2 (Nrf2) and its downstream antioxidant genes can reduce apoptosis and oxidative damage, improve the wound condition of diabetic ulcers that are not easy to heal, and have a significant role in promoting the healing of diabetic wounds [16, 17]. Diabetic foot treatment is difficult, the treatment cycle is long, the cost is high, the prognosis is poor, and it brings a heavy burden to patients and society. The traditional treatment method uses multiple debridements and dressing changes, and the wound is repaired with autologous skin grafting or flap after the wound granulation tissue grows well. However, it has a longer cycle, and a high risk of infection during treatment delays the optimal timing of treatment.

In some cases, the condition can progress to cause infections such as abscesses or osteomyelitis [18]. Infection in the skin graft area, aging of granulation buds, etc. are not conducive to the survival of the transplanted skin pieces. The incidence of damage deformities such as cosmetic depression after traditional treatment wound healing is high, bringing more inconvenience and pain to patients. Vacuum sealing drainage (VSD) treatment better solves the problems in the above traditional treatment. VSD is widely used in clinical practice as a relatively advanced surgical drainage technique. VSD can promote the increase of local neovascularization, improve local circulation and oxygen supply status, drain excessive exudate from the wound in time, reduce tissue edema, and alleviate wound infection [19]. VSD treatment better solves the problems in the above traditional treatment. The wound is placed in a closed negative pressure state, effectively reducing the infection risk. Wound exudate and necrotic “zero aggregation” allow for a relatively clean environment in a short period. The negative pressure state of the wound can effectively improve the blood ring state of the wound and reduce tissue edema. Currently, the clinical compound yellow cedar liquid coating is mostly used for the treatment of pressure sores, soft tissue infections, and other diseases [20]. Relatively little has been reported on the treatment of diabetic foot ulcers.

This detailed study specifications of the wound area, carrion, granulation tissue, wound depth, wound cycle, pain level, and formulated standard wound healing observation indicators are through a large number of literature and guidelines. The confounding of the study was reduced through rigorous training of the operating nurses, resulting in quality control of baseline management measures for both groups of patients.

It was found that compared with patients treated with saline NPWTi by applying CPL NPWTi therapy to patients with diabetic foot ulcers, CPL NPWTi therapy significantly promotes wound healing, has an anti-inflammatory effect, reduces patient hospital stay time, and reduces patient pain. This method solves the practical clinical problems, reduces the pain of patients, reduces the wound healing treatment time of patients with diabetic foot ulcers, reduces the cost of treatment, and provides a safe and effective method for treating diabetic foot ulcers. The same idea can be found in the study put forward by Leow et al. [21]. They have applied new methods in the study, and the conclusions drawn can also support this study.

However, this study also has certain limitations, the number of cases in this study is small, the observation time is short, there is a lack of effective follow-up records, and the long-term efficacy needs to be further extended. In this study, long-term follow-up studies were conducted to observe the effect of treatment further. In addition, this study mainly examined the role of NWPTi in treating grade 2-3 diabetic foot ulcers and did not study other grades of diabetic foot. There is currently no research support on the optimal drip irrigation solution and the optimal negative pressure and drip irrigation interval time, and we are ready to further explore the above points in future research.

## Figures and Tables

**Figure 1:** Wound healing condition from the two groups of patients. (a) Wound area (cm^2^). (b) Wound symptom scores. The measurement data were expressed as mean ± standard deviation (^−^*x* ± *s*). ^∗^*P* < 0.05; ^∗∗^*P* < 0.01.

**Figure 2:** Inflammatory factor indicators from the two groups of patients. (a) PCT. (b) ESR. (c) CRP. The measurement data were expressed as mean ± standard deviation (^−^*x* ± *s*).^∗^*P* < 0.05; ^∗∗^*P* < 0.01.

**Table 1:** Comparison of general data from the two groups of patients.

Indicator	CPL NPWTi group (*n* = 30)	Normal saline NPWTi group (*n* = 30)	*χ* ^2^	*P*
Sex			0.425	0.567
Male	23 (76.7%)	21 (70%)		
Female	7 (23.3%)	9 (30%)		
Age	65.4 ± 7.00	65.57 ± 6.34	0.299	0.923
Height	170.2 ± 8.25	168.93 ± 8.96	0.100	0.571
Weight	62.33 ± 4.41	60.9 ± 5.47	0.987	0.268
Blood glucose level	11.39 ± 0.86	11.74 ± 0.90	1.000	0.124
Complication			0.919	0.705
Numb	2	1		
Pain	1	1		
Skin ulceration	2	2		
Infection	3	3		

**Table 2:** Quantitative table of diabetic foot symptoms.

Symptoms	0 points	1 point	2 points	3 points	Weight
Wound area (cm^2^)	0-4	5-8	9-12	13-16	2
Carrion	None	Small amount	Medium	Substantial	2
Granulation tissue	Heal	Red	Pale edema	The color is gray and dark	2
Wound depth	Heal	Subcutaneous tissue	Deep tendon	Deep bone	2
Creation of skin color	Normal	Reddish	Redder	Bright red and shiny	1
Swelling around the wound	None	Slight swelling	Pronounced swelling	Severe swelling	1
Temperature around the wound	Normal	Slightly hot	Hotter	Hot	1
Pain	None	Mild	Moderate	Severe	1

Note: the wound area is traced using a transparent checkerboard, and the Image J image processing software calculates the size. Determination of the amount of carrion: based on the wound area occupied, it is divided into no (0), a small amount (<25%), medium amount (25% to 50), and a large amount (≥50%). Pain levels are assessed using a pain visual simulation scale.

**Table 3:** Comparison of wound healing conditions from the two groups of patients.

Indicator	Normal saline NPWTi group (*n* = 30)	CPL NPWTi group (*n* = 30)	*χ* ^2^	*P*
Before treatment				
Wound area(cm^2^)	9.263 ± 1.619	9.212 ± 1.991	0.831	0.914
Wound symptom scores	19.833 ± 2.479	20.333 ± 1.807	0.996	0.376
Treatment for 10 days				
Wound area (cm^2^)	5.566 ± 1.518	8.146 ± 1.644	0.961	0.309
Wound symptom scores	17.600 ± 1.905	16.500 ± 2.177	0.991	0.042
Treatment for 20 days				
Wound area (cm^2^)	6.461 ± 1.328	5.663 ± 1.708	0.889	0.048
Wound symptom scores	12.367 ± 1.328	10.633 ± 2.109	0.859	0.002
Treatment for 30 days				
Wound area (cm^2^)	4.874 ± 1.725	2.446 ± 1.365	0.004	<0.001
Wound symptom scores	6.933 ± 1.337	5.5 ± 1.503	0.920	<0.001

**Table 4:** Comparison of inflammatory factor indicators from the two groups of patients.

Inflammatory factor indicators	CPL NPWTi group (*n* = 30)	Normal saline NPWTi group (*n* = 30)	*χ* ^2^	*P*
Before treatment				
PCT	0.358 ± 0.061	0.35 ± 0.074	0.642	0.596
ESR	28.789 ± 1.931	29.218 ± 2.224	0.577	0.428
CRP	25.533 ± +6.458	25.400 ± 6.200	3.261	0.258
Treatment for 10 days				
PCT	0.211 ± 0.049	0.248 ± 0.058	1.233	0.011
ESR	24.366 ± 1.634	25.517 ± 2.262	1.402	0.254
CRP	16.300 ± 2.493	18.2 ± 3.478	0.403	0.018
Treatment for 20 days				
PCT	0.097 ± 0.029	0.129 ± 0.041	0.993	0.001
ESR	20.997 ± 1.935	19.748 ± 2.049	0.997	0.018
CRP	5.333 ± 1.093	6.433 ± 1.888	0.967	0.008
Treatment for 30 days				
PCT	0.075 ± 0.029	0.102 ± 0.027	1.411	<0.001
ESR	17.681 ± 1.458	16.634 ± 1.399	0.999	0.006
CRP	4.500 ± 0.900	5.5 ± 1.570	0.805	0.003

**Table 5:** Comparison of positive bacterial culture from the two groups of patients.

Positive bacterial culture	CPL NPWTi group (*n* = 30)	Normal saline NPWTi group (*n* = 30)	*χ* ^2^	*P*			
Before treatment	29 (96.67%)	30 (100%)	1.113	0.321			
Treatment for 10 days	18 (60%)	23 (76%)	0.981	0.034			
Treatment for 20 days	8 (26.6%)	19 (63.3%)	0.962	0.008			
Treatment for 30 days	6 (20%)	16 (53.3%)	0.989	0.007			

**Table 6:** Comparison of number of days in hospital and from the two groups of patients.

Indicator	CPL NPWTi group (*n* = 30)	Normal saline NPWTi group (*n* = 30)	*χ* ^2^	*P*			
Number of days in hospital	27.2 ± 8.3	39.1 ± 15.2	-0.572	<0.001			
Pain scores during dressing change	2.7 ± 1.4	3.9 ± 2.5	-3.466	0.015			

## Data Availability

The datasets used and analyzed during the current study are available from the corresponding author upon reasonable request.
